The article "Ointment of Brassica oleracea var. capitata Matures the Extracellular Matrix in Skin Wounds of Wistar Rats" was retracted in 2025. Reasons: duplicated images; overlap with earlier publications; unreliable results or conclusions; concerns about the images.

# Ointment of *Brassica oleracea* var. *capitata* Matures the Extracellular Matrix in Skin Wounds of Wistar Rats

**DOI:** 10.1155/2015/919342

**Published:** 2015-06-11

**Authors:** Mariáurea Matias Sarandy, Rômulo Dias Novaes, Sérgio Luiz Pinto da Matta, Jose Mario da Silveira Mezencio, Marcelo Barreto da Silva, José Cola Zanuncio, Reggiani Vilela Gonçalves

**Affiliations:** ^1^Department of General Biology, Federal University of Viçosa, 36570-000 Viçosa, MG, Brazil; ^2^Department of Structural Biology, Federal University of Alfenas, 37130-000 Alfenas, MG, Brazil; ^3^North University Center of the Espirito Santo, Federal University of Espirito Santo, 29932-540 São Mateus, ES, Brazil; ^4^Department of Entomology, Federal University of Viçosa, 36570-000 Viçosa, MG, Brazil; ^5^Department of Animal Biology, Federal University of Viçosa, 36570-000 Viçosa, MG, Brazil

## Abstract

Wound healing is a complex process that aims to restore damaged tissue. Phytotherapeutics, such as cabbage, *Brassica oleracea* var. *capitata* (Brassicaceae), and sunflower, *Helianthus annuus* L. (Asteraceae) oil, are used as wound healers. Five circular wounds, each 12 mm in diameter, were made in the dorsolateral region of each rat. The animals were divided into four groups: balsam (*B. oleracea*); ointment (*B. oleracea*); sunflower oil (*Helianthus annuus*); control (saline solution 0.9%). These products were applied daily for 20 days and every four days the tissues of different wounds were removed. The wound contraction area, total collagen, types I and III collagen, glycosaminoglycans, and tissue cellularity were analyzed. In the groups that received ointment and balsam there was reduction in the wound area on days 4, 8, 12, and 20. Throughout the trial period, the balsam and ointment groups showed a higher amount of total collagen, type I collagen, and glycosaminoglycan compared to the others groups. The rats in the groups treated with *B. oleracea* var. *capitata* showed a higher number of cells on days 8, 16, and 20. *B. oleracea* was effective in stimulating the maturation of collagen and increasing the cellularity, as also in improving the mechanical resistance of the newly formed tissue.

## 1. Introduction

Wound repair is a process that involves cellular and extracellular mechanisms, which aim to attain cell proliferation and vascularization of the injured tissue. The increase in cell number is because of the recruitment of inflammatory cells that secrete cytokines and attract others cells to the lesion site [1]. Mediators are also released to stimulate neovascularization and improve nutrition and tissue oxygenation [2, 3]. This dynamic repair process is divided into three phases: inflammation, proliferation, and maturation. In the early stages, in addition to leukocytes, the number of fibroblasts and vessels increase and a large amount of type III collagen and glycosaminoglycans is observed, forming a weaker tissue called granulation tissue, which is more susceptible to severance [4]. In the final phase of repair, the amount of sulfated components decreases and type III collagen is replaced by thicker and stronger type I collagen [5]. A proper synthesis of the different components of the matrix is required for the process to take place smoothly and to ensure strength and resistance to the tissue [4, 6].

The effects of cabbage* Brassica oleracea* L. (Brassicaceae) and sunflower* Helianthus annuus* L. (Asteraceae) on wound healing are still unclear. Cabbage has high nutritional value [7] and is a source of anticancer glucosinolates [8]. In addition, it also has antimicrobial and antioxidant properties [9] and has high levels of flavonoids [8] and anthocyanins [10], with an anti-inflammatory and protecting power of the new-formed tissue, protecting the free radical action and increasing the levels of antioxidant enzymes [11] and pectin [12]. The action in the reduction of oxidative stress may be linked to the stimulation of a pathway known as Nrf2, a key protein for induction of antioxidant agents [13].

Treatment of human diseases with natural extracts and oils is increasing constantly [14–16]. These products have been used for the development of new drugs and have shown a promising therapy [17].* Helianthus annuus* oil, with medium-chain triglycerides and essential fatty acids, has been used to stimulate cellular nutrition, tissue regeneration, and wound healing [16].

The aim of this study is to evaluate the reduction of the wound area, reconstitution of the extracellular matrix, and cell proliferation of the cutaneous scar tissue of Wistar rats* Rattus norvegicus* Berkenhout, 1769 (Rodentia: Murinae), treated with ointment and balsam of cabbage* Brassica oleracea* var.* capitata* (Brassicaceae) extract.

## 2. Materials and Methods

### 2.1. Experimental Site

The experiment was carried out in the “Laboratório de Nutrição Experimental” of the “Departamento de Nutrição” of the “Universidade Federal de Viçosa” (UFV) in Viçosa, Minas Gerais State, Brazil.

### 2.2. Animals

Thirty-two male Wistar rats (*R. norvegicus*) (302.23 ± 26.23 g) of 60 days of age were obtained from the “Biotério Central da Universidade Federal de Viçosa” in Viçosa, Minas Gerais State, Brazil. These rodents were individualized in clean cages and maintained at 22 ± 2°C, with 65 ± 5% relative humidity, and a 12-hour light/dark cycle. Food and water were provided* ad libitum*. The experiment was approved by the Animal Ethics Committee of the Universidade Vale do Rio Doce (Univale) (registration: 18/2002).

### 2.3. Formulation of the Products Tested

*B. oleracea* var.* capitata* leaves were collected, sanitized by immersion in 2% sodium hypochlorite in distilled water during 2 minutes, and washed into autoclaved drinking water for 2 minutes. The leaves were macerated adding ethanol/propylene glycol (4 : 1 v.v) as extracting solvent. Then, the suspension was subjected to ultrasonication (Unique, MaxiClean 1400, São Paulo, SP) and vacuum filtration and the concentrated extract was heated at 55°C in an oven for 24 h to remove the solvent. Finely, the extract was incorporated into the ointment base and balsam base until complete homogenization. The formulations investigated were prepared as follows:* Balsam*:* B. oleracea* var.* capitata* glycolic extract (10 wt.%), preservatives (methylparaben, propylparaben, and butylated hydroxytoluene [1 : 1, 30 wt.%]), oils (hydrogenated castor oil, triglycerides of caprylic acid, capric acid, caproic acid, and lauric acid [1 : 1, 20 wt.%]), and demineralized water (40 wt.%) [18];* ointment*:* B. oleracea* var.* capitata* glycolic extract (10 wt.%), cetostearyl alcohol (5 wt.%), ethoxylated sorbitan monooleate (10 wt.%), Vaseline (10 wt.%), fatty acid with polyol ester (5 wt.%), anhydrous lanolin (15 wt.%), carbamide (5 wt.%), preservatives (methylparaben, propylparaben, and butylated hydroxytoluene [1 : 1, 10 wt.%]), hydrogenated castor oil (5 wt.%), and demineralized water (15 wt.%) [18];* sunflower oil* (*H. annuus*): medium-chain triglyceride oil (caprylic acid, capric acid, caproic acid, and lauric acid [80 wt.%]) and essential fatty acids (linoleic acid [20 wt.%]), in a ratio of 1 : 1 (purchased from Saniplan Essential Products, Rio de Janeiro, RJ, Brazil).

### 2.4. Experimental Design

Prior to creating the wound, the animals were anesthetized by intramuscular injection of ketamine (50 mg/kg) and xylazine (20 mg/kg). Dorsolateral shaving of the animals was performed, and the area was degreased with ethyl ether (Merck, Rio de Janeiro, Brazil), followed by the use of 70% ethanol and 10% povidone-iodine for antisepsis (Johnson Diversey; Rio de Janeiro, Brazil). Three circular wounds, 12 mm in diameter, for secondary intention wound closure, were made by surgical incision in the skin and the subcutaneous cell tissue with a scalpel until the dorsal muscular fascia was exposed [19]. The animals were randomized into four groups with 8 animals in each group: balsam (*B. oleracea* var.* capitata*); ointment (*B. oleracea* var.* capitata*); sunflower oil (*H. annuus*); and control (saline solution at 0.9%). The wounds were treated with 0.6 g of ointment and balsam once a day for 20 days. Treatments were started immediately after surgery and repeated daily. The fragments containing the center and the edges of the wounds were harvested every 4 days.

### 2.5. Progression of the Closure of Wounds

The closure of the wounds was evaluated in an area every 4 days by taking images with a digital camera W30, Sony, Tokyo, Japan, of 320 × 240 pixels (24 bits/pixel). The wound area was calculated by computerized planimetry, using the Image Pro-Plus software, version 4.5 (Media Cybernetics, Silver Spring), previously calibrated. The wound contraction index was calculated using the following formula: Initial wound area (*A*_0_) − wound area on day (*A*_*i*_) ÷ initial wound area × 100 [20]. The healing process was analyzed in the sample collected on the last day of the experiment.

### 2.6. Histological Processing

The fragments of the wound were removed every four days and fixed in formaldehyde at 10%, dehydrated in ethanol, diaphonized with xylene, and embedded in paraffin. Cuts, 4 *μ*m thick, were obtained with a Reichert-Jung 2045 Multicut Rotary Microtome (Germany), using 1 from every 20 sections to avoid repetition of the studied area. The sections were stained with hematoxylin and eosin (H&E) for analysis of cells and blood vessels and to differentiate the collagen fibers, which were stained with Sirius Red (Sirius F3B Red, Mobay Chemical Co., Union, New Jersey, USA) and observed under polarized light microscopy (Sigma, Saint Louis, Missouri, USA) [19].

The animals were weighed every 4 days, an interval coinciding with the removal of wound fragments. The fragments that were removed for histological analysis were preserved in 10% buffered formaldehyde for 24 hours. The material was processed for paraffin embedding by ethanol dehydration, diaphonization with xylene, infiltration, and embedding in paraffin wax. Cuts of 4 *μ*m were obtained with a rotary microtome (Reichert-Jung 2045 Multicut, Germany) and stained with Picrosirius (Sirius Red F3B, Mobay Chemical Co., Union, New Jersey, USA).

Images of the histological sections were captured with a polarization microscope (Olympus AX-70, Brazil), and the amounts of type I and III collagen fibers were evaluated. Four random images from different parts of the field were obtained from each sample, for a total tissue area of 5.37 × 106 *μ*m^2^. A grid containing 300 points in a test area of 73 × 10^3^ *μ*m^2^ was superimposed on each image for this analysis. The stereological parameters of volume density (*V*_*v*_) were calculated by the count of points on fibroblasts, total collagen fibers, and collagen types I and III, using the index *V*_*v*_ = *P*_*p*_/*P*_*t*_, in which *P*_*p*_ was the number of points occurring over the structure of interest and *P*_*t*_ is the total number of points on the test system [18]. The collagen fibers were analyzed according to their properties of birefringence under polarization. The intervals defining the identification of the colors red, green, and black were previously standardized and then used for all images obtained. Red represented type I collagen fibers, green, type III collagen fibers [19], and black, the regions where no fibers were found. The program provided the percentage of the area corresponding to each color.

### 2.7. Total Collagen Analysis and Glycosaminoglycans

Thirty-five sections, 8 *μ*m thick, were stained with Sirius Red and Fast Green to quantify the levels of collagen and total protein, using the spectrophotometric method described previously [18]. In this method, the maximum absorbance of the Sirius Red (540 nm) and Fast Green (605 nm) dyes corresponded to the amount of total collagen and noncollagenous proteins, respectively. For each section used in the collagen analysis, a corresponding serial section was obtained; which was used for the analysis of glycosaminoglycans. The tissue content of glycosaminoglycan was determined by the method of Corne [21], modified. The sections were immediately transferred to 10 mL of 0.1% (w/v) Alcian blue 8GX solution (0.16 M sucrose solution buffered with 0.05 mL sodium acetate at pH 5.0). After successive rinses in 10 mL of a 0.25 M sucrose solution, the dye that adhered to the tissue was extracted with 10 mL of 0.5 M magnesium chloride, and the absorbance of the resultant solution was analyzed in a spectrophotometer at 580 nm.

### 2.8. Cellularity

To determine tissue cellularity, 50 histological fields from each group (40x objective lens) were randomly sampled, with a total area of 3.65 × 10^4^ *μ*m^2^. To avoid repeated analysis of the same histological area, the sections were evaluated in a semiseries, using 1 in every 20 sections. Computer-based image analysis was used to determine the cell number in the scar tissue. Digital images (Figures 2(a) and 2(b)) were prepared using the Image Pro-Plus 4.5 software (Media Cybernetics, Silver Springs, MD, USA) and the distribution of the cell nuclei was determined as follows: (a) Scar tissue was segmented in a pure black and white image, (b) the cell nuclei were selected and assigned a white color, (c) the remaining tissue was selected and assigned a black color, and (d) the number of cell nuclei (represented by white points) in the whole image was automatically measured by the program [18].

### 2.9. Statistical Analysis

The normality of distribution of the data was verified by the Shapiro-Wilk test. The data were submitted to the Kruskal-Wallis test (*p* < 0.05) with the Sigma Stat3.0 software (Systat Software Inc., Chicago, Illinois, USA).

## 3. Results

### 3.1. Wound Contraction

The wound contraction index was higher on the 4 and 16 days in the groups treated with balsam and ointment of* B. oleracea* var.* capitata* than in the other groups. On the 4 and 16 days, reductions in the size of the wound were also greater in the groups treated with* B. oleracea* than* H. annuus* and the control group. All wounds were completely healed on day 20 (Table 1).

### 3.2. Production of Collagen and Glycosaminoglycans

The levels of total collagen and glycosaminoglycans were similar in tissues without lesions in all treatments (Table 2). On days 8, 16, and 20, the total collagen content was higher with balsam and ointment (*B. oleracea* var.* capitata*) than in the control and sunflower groups; however, on day 20 the balsam group (*B. oleracea* var.* capitata*) had a greater amount of collagen than the sunflower oil group (*H. annuus*) (*p* < 0.05). On days 8, 12, 16, and 20, the glycosaminoglycan content was higher in the groups treated with* B. oleracea* var.* capitata*. At the end of the experiment, the glycosaminoglycans index was lower in the groups treated with* B. oleracea* var.* capitata* (day 20, Table 2).

### 3.3. Types I and III Collagen Fibers

On days 4, 8, 12, 16, and 20, the number of fibers in type III was higher in the groups treated with balsam and ointment* B. oleracea* var.* capitata* (Table 3). On the days 8, 16, and 20, the balsam and ointment groups showed a greater number of type I fibers compared to the other groups (*p* < 0.05) (Table 4). These data could be confirmed from the analysis in Figure 1, which shows the predominance of type I collagen (red fibers) in the balsam and ointment groups after 20 days of treatment (Figure 1).

### 3.4. Cellularity and Blood Vessels

The number of cells in the groups treated with balsam and ointment (*B. oleracea* var.* capitata*) increased on days 16 and 20 compared to the* H. annuus* and control groups (Figures 2(c) and 3). After analysis of Figure 2(a) increased density of blood vessels was observed mainly in the balsam group compared to the other groups.

## 4. Discussion

The area and the wound contraction index showed the best results in the groups receiving treatment with* B. oleracea*, indicating the action of this herbal medicine in cell proliferation and differentiation. In this process it is important to highlight the activation of chemical mediators that promoted the differentiation of fibroblasts into myofibroblasts [22, 23]. The activity of these cells was demonstrated with other treatments such as the herbal ointment* Jasminum grandiflorum* Linn. (Oleaceae), which was obtained at different concentrations, with a greater contraction rate of the wounds under the action of myofibroblasts, at 14 days [24]. The use of medicinal plants stimulates the production of connective and epithelial tissues that are important to form the framework and promote wound closure [16, 25]. The area and the wound closing speed are important for healing, as they serve as markers to observe the evolution of the wound [26]. The smaller area and the fastest speed of wound contraction in the groups treated with balm and* B. oleracea* ointment indicate the action of its components in cell proliferation and differentiation.

Groups of rats that were treated with* B. oleracea* showed high total collagen, similar to that found for* Ganoderma lucidum* (M. A. Curtis:Fr.) P. Karst, a popular medicinal mushroom, rich in flavonoids and phenols, a compound also present in* B. oleracea* [26–28]. This compound is responsible for therapeutic effects, such as antioxidant, anti-inflammatory, and antifungal effect, and also known to promote quick healing because of its antimicrobial properties that promote complete collagen synthesis [28, 29]. Experiments in* Jasminum grandiflorum* ointment extract showed an increase in the amount of hydroxyproline in the granulation tissue. This is an important amino acid for collagen production and consequently of extracellular matrix [24]. In addition, treatment with Jatyadi Taila (oil) increased the total protein levels in Wistar rats during skin repair [30].

The lowest content of glycosaminoglycans and collagen increased in the groups treated with* B. oleracea* at the end of experiment, which demonstrated that mature tissue was acquired during the treatment, as the less sulfated array was the greatest resistance to the newly formed tissue. These data agreed with the results observed in rats treated with* Annona squamosa* L. extract [Annonaceae]. This herbal ointment promoted the increase of glycosaminoglycans at the beginning and end of the reduction treatment, which helped in regulation, proliferation, migration, and differentiation during tissue repair [31]. Molecules, such as sulfated glycosaminoglycans, attracted water and helped cell migration, predominantly during the formation of granulation tissue and allowed an efficient and rapid inflammatory process [32, 33]. Moreover, these molecules served as a support for the formation of the first collagen (collagen type III), having in its structure myofibrils, with an absence of covalent bonds, which were produced quickly by fibroblasts [22]. At the end of the healing process, the glycosaminoglycans decreased and the total collagen increased, because at this stage the tissue needed stability and strength [34]. Analysis of the total collagen was important to observe the wound strength and the collagen maturation index (CMI) was a common parameter to analyze the maturation of the scar [5].

The largest number of type III collagen fibers at the beginning of treatment with* B. oleracea* demonstrated the importance of this constituent in the formation of granulation tissue; and reduction of these fibers after the treatment showed the effectiveness of the herbal formation of more resistant fabrications. These results were similar to those found in the extract of* Bathysa cuspidata*, where there was an increase in collagen III the seventh and fourteenth days and it decreased after 21 days of treating the skin wounds in Wistar rats [35].* B. oleracea* has stimulated cell proliferation, protein synthesis, and tissue remodeling in different types of lesions [12]. Collagen III, the main constituent of the granulation tissue, was being replaced by collagen I, rich in covalent bonds, during the repair process. This enabled organization in bundles of fibers that formed new tissues, stronger and resistant [2].* B. oleracea* treatment caused a steady increase in the amount of type I collagen fibers showing a higher percentage at the end of the experiment, similar to that observed in rats treated with olive oil, which stimulated collagen deposition and, hence, the resistance of the healing [17]. The herbal medicine stimulated the synthesis of collagen I, producing a strong and tough scar with high levels of BMI, indicating the predominance of type I collagen on type III collagen. Alternative treatments such as laser therapy, with high doses of energy efficiency, were shown to stimulate the production of collagen type I [18, 36]. Studies with propranolol, for 21 days, in rats, demonstrated the presence of type I collagen fibers that were thicker and reddish [22]. However, the synthesis of this component of the matrix was connected to good tissue vascularization that provided oxygen and nutrients to the tissue for optimal metabolic activity of the fibroblasts and was more abundant and important for cell synthesis of the matrix components [2, 37, 38]. In addition to flavonoids, the compounds and phytochemicals in the* B. oleracea* extract included phenols, sulforanos, and anthocyanins [27, 28, 39], which had a positive effect on collagen type I expression and gradually influenced a reduction in the expression of collagen type III [28].

The increase of cells in the wounds of animals treated with* B. oleracea* was related to the process of cell migration mediated by cytokines and growth factors, such as the application of propolis in mice, which demonstrated its anti-inflammatory effect, with an increase in neutrophils and macrophages [40]. The topical use of olive oil with oleic acid and phenolic compounds accelerated the inflammatory process cell migration increasing the neutrophil, macrophage, and cytokine production [17, 41]. Cells present in the inflammatory infiltrate synthesized chemical mediators that promoted neoangiogenesis and cell migration, increasing the share of defense systems and stimulating matrix synthesis [38]. The cellularity found in most tissues was removed from groups of mice treated with* B. oleracea*, which indicated an efficient repair process, and other brassicas, such as broccoli, presented sulforanos that inhibited important pathways to inflammation [42]. In inflammatory cells, fibroblasts, vascular cells that synthesized cellular mediators, and all components of the extracellular matrix had to be highlighted [27]. In this context,* Angelica sinensis* extract [42], diet with* Centella asiatica* L. [Apiaceae] [43], and* Marrubium vulgare* [horehound], Lamiaceae [44], rich in anthocyanins, had anti-inflammatory and antioxidant activities, which were suitable for essential skin repair. This cellularity that was directly linked to tissue vascularization was observed in the group treated with* B. oleracea*. The formation of new vessels is responsible for distribution of oxygen and nutrients in the cells recruited, mainly, in the tissues newly formed providing a better healing [25]. These data can be demonstrated through the analysis of tissues of rats that received olive oil application [17] and male albino rats that received topical ointment of the* J. grandiflorum* extract [24]. Tissue repair resulted from the catabolic and anabolic reactions repeated by different cell types, and hence, the increased cellularity indicated that the repair process was successful in reestablishing homeostasis and scar formation [26].

The ointment and balsam of* B. oleracea* were effective in accelerating the wound closure procedure and in forming a basis for the formation of granulation tissue and mature scar tissue, rich in type I collagen. These findings demonstrated that* B. oleracea* might modulate the repair of skin wounds in the initial and final stages of the healing process.

## Figures and Tables

**Figure 1:** Photomicrographs of the scar tissue on days 0, 4, 8, 16, and 20 of the experiment (Sirius Red staining; bar = 60 *μ*m). Tissues were collected every 4 days for 20 days of treatment. Balsam:* Brassica oleracea* oil; ointment:* Brassica oleracea* lanolin; sunflower:* Helianthus annuus* oil; control: 0.9% saline solution.

**Figure 2:** Cellularity in scar tissue of rats treated with* Brassica oleracea* and* Helianthus annuus*. The top panels (a and b) are representative photomicrographs of the computational method of color segmentation to estimate cell distribution in scar tissue (c). Digital images of skin sections stained with hematoxylin and eosin (a, bar = 40 *μ*m) were computationally modified using a color-cube-based mode and a new mask was applied by selecting all pixels of varying dark blue color levels. Then, a new image in black and white was generated after color segmentation (b, bar = 40 *μ*m) and the number of cell nuclei (white color) was measured by point counting. Balsam:* Brassica oleracea* oil; ointment:* Brassica oleracea* lanolin; sunflower:* Helianthus annuus* oil; control: 0.9% saline solution. Data are represented as mean and standard deviation (mean ± SD). *∗* denotes statistical differences between groups (*p* < 0.05), *∗* versus control; Kruskal-Wallis test.

**Figure 3:** Representative photomicrographs of tissue cellularity in skin sections of rats observed under light microscope (H&E staining, bars = 25 *μ*m). Tissue fragments were collected from different wounds on days 0, 4, 8, 16, and 20 days. Balsam:* Brassica oleracea* oil; ointment:* Brassica oleracea* lanolin; sunflower:* Helianthus annuus* oil; control: 0.9% saline solution.

**Table 1:** Effects of *Brassica oleracea* (balsam and ointment) and *Helianthus annuus* (sunflower oil) on the area and the rate of wound contraction in rats evaluated every 4 days for 20 days of treatment.

Day	Area/contraction	Balsam	Ointment	Sunflower	Control
0	*A* (mm^2^)	121.35 ± 1.11	122.23 ± 1.06	120.56 ± 1.77	120.67 ± 1.99
	WCI (%)	0.00 ± 0.00	0.00 ± 0.00	0.00 ± 0.00	0.00 ± 0.00

4	*A* (mm^2^)	109.85 ± 5.43^*∗*†^	109.54 ± 3.32^*∗*†^	118.18 ± 4.32	117.46 ± 2.54
	WCI (%)	9.47 ± 2.02^*∗*†^	10.12 ± 2.32^*∗*†^	1.967 ± 1.28	2.66 ± 1.42

8	*A* (mm^2^)	75.15 ± 4.32^*∗*^	65.76 ± 7.14^*∗*^	78.32 ± 3.23^*∗*^	88.87 ± 5.43
	WCI (%)	38.07 ± 4.56^*∗*^	46.19 ± 5.45^*∗*^	35.03 ± 4.31^*∗*^	26.35 ± 4.20

12	*A* (mm^2^)	42.76 ± 6.32^*∗*^	42.56 ± 5.54^*∗*^	50.46 ± 4.55^*∗*^	60.65 ± 4.65
	WCI (%)	56.52 ± 5.43	65.18 ± 5.43^*∗*^	58.14 ± 4.98^*∗*^	49.73 ± 5.21

16	*A* (mm^2^)	10.13 ± 3.13^*∗*†^	8.33 ± 4.32^*∗*†^	17.65 ± 3.12	20.32 ± 6.32
	WCI (%)	91.65 ± 4.87^*∗*^	90.18 ± 4.79^*∗*^	85.36 ± 4.43	83.16 ± 4.43

20	*A* (mm^2^)	0.00 ± 0.00	0.00 ± 0.00	0.00 ± 0.00	0.00 ± 0.00
	WCI (%)	100.00 ± 0.00	100.00 ± 0.00	100.00 ± 0.00	100.00 ± 0.00

Data are reported as mean ± S.D. *A*: wound area, WCI: wound contraction index; balsam: *Brassica oleracea* oil; ointment: *Brassica oleracea* lanolin; sunflower oil: *Helianthus annuus;* control: 0.9% saline; ^*∗*^ *p* < 0.05, statistically different compared to the control group; ^†^ *p* < 0.05, statistically different compared to sunflower oil. Kruskal-Wallis test.

**Table 2:** Levels of total collagen and glycosaminoglycans in the scar tissue of rats treated with *Brassica oleracea* (balsam and ointment) and *Helianthus annuus* (sunflower oil) and evaluated every 4 days for 20 days of treatment.

Treatments	Day 0	Day 4	Day 8	Day 12	Day 16	Day 20
Collagen (*µ*g/g protein)						
Balsam	512.11 ± 46.13	200.34 ± 43.23	277.63 ± 30.81^*∗*^	305.23 ± 27.23	594.58 ± 9.07^*∗*^	493.09 ± 5.70^*∗*†^
Ointment	502.45 ± 39.32	201.23 ± 46.45	299.53 ± 33.27^*∗*^	310.45 ± 32.43	581.66 ± 34.33^*∗*^	421.82 ± 54.11^*∗*^
Sunflower	512.26 ± 50.25	200.34 ± 44.32	210.42 ± 42.22	315.35 ± 36.32	519.28 ± 42.82	402.17 ± 29.16
Control	510.25 ± 59.24	199.43 ± 45.32	203.72 ± 51.03	301.34 ± 34.67	520.47 ± 43.91	400.34 ± 32.14

Glycosaminoglycans (*µ*g/g protein)						
Balsam	39.46 ± 7.33	52.34 ± 6.23	88.52 ± 10.62^*∗*^	70.43 ± 7.23^*∗*^	71.23 ± 8.18^*∗*^	47.36 ± 9.02^*∗*†^
Ointment	37.28 ± 8.07	51.34 ± 5.32	75.23 ± 8.30^*∗*^	73.23 ± 8.34^*∗*^	66.80 ± 10.37^*∗*^	42.25 ± 8.16^*∗*^
Sunflower	39.36 ± 6.52	53.45 ± 5.23	59.21 ± 8.25	59.55 ± 7.32	60.00 ± 7.54	56.51 ± 6.10
Control	40.35 ± 5.12	50.72 ± 5.23	58.11 ± 9.05	59.20 ± 6.23	60.19 ± 7.54	56.51 ± 6.10

Balsam: *Brassica oleracea*, oil; ointment: *Brassica oleracea* lanolin; sunflower oil: *Helianthus annuus*; control: 0.9% saline; ^*∗*^ *p* < 0.05 denotes a statistical difference compared to the control group; ^†^ *p* < 0.05 denotes a statistical difference compared to the sunflower oil group. Day 0 represents the unharmed tissue. Data are represented as mean and standard deviation (mean ± S.D.). Kruskal-Wallis test.

**Table 3:** Proportion of type I collagen fibers in scar tissue of rats receiving *Brassica oleracea* (balsam and ointment) and *Helianthus annuus* (sunflower oil) evaluated every 4 days for 20 days of treatment.

Treatments	Type I collagen fibers					
	Day 0	Day 4	Day 8	Day 12	Day 16	Day 20
Balsam	24.45 ± 10.01	7.83 ± 0.39^*∗*^	14.23 ± 0.47^*∗*†^	18.17 ± 0.45^*∗*^	21.62 ± 1.82^*∗*†^	39.95 ± 3.23^*∗*†^
Ointment	27.55 ± 12.62	7.19 ± 0.78^*∗*^	15.14 ± 0.49^*∗*†^	17.53 ± 0.56^*∗*^	21.45 ± 1.73^*∗*†^	30.76 ± 3.52^*∗*†^
Sunflower	25.99 ± 14.78	6.27 ± 0.87^*∗*^	7.36 ± 0.78^*∗*^	15.58 ± 1.33^*∗*^	17.12 ± 1.71^*∗*^	21.70 ± 4.71^*∗*^
Control	25.88 ± 13.82	2.69 ± 0.58	3.68 ± 0.46	7.26 ± 0.70	9.40 ± 0.57	11.20 ± 4.71

Balsam: *Brassica oleracea* oil; ointment: *Brassica oleracea* lanolin; sunflower oil: *Helianthus annuus*; control: 0.9% saline; ^*∗*^ *p* < 0.05, statistically different compared to the control group; ^†^ *p* < 0.05, statistically different compared to the sunflower oil. Day 0 represents the unharmed tissue. Data are represented as mean and standard deviation (mean ± S.D.). Kruskal-Wallis test.

**Table 4:** Proportion of type III collagen fibers in scar tissue of rats receiving *Brassica oleracea* and sunflower oil evaluated every 4 days for 20 days of treatment.

Treatments	Type III collagen fibers					
	Day 0	Day 4	Day 8	Day 12	Day 16	Day 20
Balsam	8.90 ± 0.51	43.39 ± 0.77^*∗*†^	42.23 ± 1.21^*∗*†^	35.53 ± 0.91^*∗*†^	28.62 ± 0.82^*∗*†^	19.95 ± 0.53^*∗*†^
Ointment	8.55 ± 0.52	43.19 ± 1.01^*∗*†^	42.56 ± 0.95^*∗*†^	34.23 ± 0.56^*∗*†^	22.24 ± 0.54^*∗*^	18.76 ± 0.52^*∗*†^
Sunflower	8.73 ± 0.44	21.71 ± 0.76	23.71 ± 1.00^*∗*^	20.13 ± 0.73^*∗*^	20.12 ± 1.71^*∗*^	11.70 ± 1.01^*∗*^
Sal	8.82 ± 0.45	20.57 ± 0.66	21.68 ± 0.76	16.92 ± 0.49	13.06 ± 0.69	11.85 ± 0.611

Balsam: *Brassica oleracea* oil; ointment: *Brassica oleracea* lanolin; sunflower oil: medium-chain triglycerides and linoleic acid; Sal: control, 0.9% saline; ^*∗*^ *p* < 0.05, statistically different compared to the control group; ^†^ *p* < 0.05, statistically different compared to the sunflower oil. Day 0 represents the unharmed tissue. Data are represented as mean and standard deviation (mean ± S.D.). Kruskal-Wallis test.
